The article "Construction and Empirical Study of Nursing Quality Evaluation Index System of Hepatobiliary Surgery Based on ERAS Concept" was retracted in 2022. Reason: concerns about the peer review.

# Construction and Empirical Study of Nursing Quality Evaluation Index System of Hepatobiliary Surgery Based on ERAS Concept

**DOI:** 10.1155/2022/1117880

**Published:** 2022-04-14

**Authors:** Zengfen Pang, Xingli Wang, Yanfang Wu, Huan Zhang, Amei Huang, Xianghong Li

**Affiliations:** ^1^Department of Surgery, Cancer Hospital of Shandong First Medical University, Jinan, 250117 Shandong, China; ^2^Department of Care, Cancer Hospital of Shandong First Medical University, Jinan, 250117 Shandong, China; ^3^Department of Hepatobiliary Surgery, Yantaishan Hospital, Yantai, 264000 Shandong, China; ^4^Proton Center, Cancer Hospital of Shandong First Medical University, Jinan, 250117 Shandong, China; ^5^Hepatobiliary and Osseous Soft Areas of the First Affiliated Cancer Hospital of Shandong Medical University, Jinan, 250117 Shandong, China

## Abstract

**Objective:**

To study the index system of enhanced recovery after surgery (ERAS) nursing evaluation, as a basis for the quality evaluation of hepatobiliary care, continue to improve the quality of hepatobiliary care.

**Methods:**

The 300 cases of hepatobiliary surgical diseases treated in our hospital from January 2019 to December 2020 were randomly selected as the subjects of this study. Through clinical trials, two groups of subjects were used, one for the ERAS care group and the traditional care group. Through the questionnaire survey and access to the relevant research data, statistical data analysis was performed using the SPSS 22.0 software. Metrics were analyzed as descriptive by mean, standard deviation, and coefficient of variation. The Visual Analogue Score (VAS) Hepatobiliary Surgery Nursing Service evaluation form, service evaluation form, postoperative incidence of adverse reaction rate, patient satisfaction, and readmission rate questionnaire were established from the aspects of structural quality and process quality. An index system of hepatobiliary surgery nursing quality evaluation based on the ERAS concept was constructed.

**Results:**

This study compared the degree of VAS pain through postoperative care. The ERAS care group scored significantly lower than in the traditional care group. Nursing patients based on ERAS are very satisfied with the quality of care services. By comparing patient postoperative adverse reactions, satisfaction, and readmission rates, the ERAS care group was significantly better than the traditional care group. It can be seen that a good nursing quality evaluation index system can truly and objectively reflect the level of nursing quality and promote the hospital to further improve the medical quality.

**Conclusion:**

The research on the construction of nursing quality evaluation index system of hepatobiliary surgery based on ERAS concept provides a more scientific evaluation standard for nursing quality evaluation of hepatobiliary surgery ERAS, creates conditions for digital and intelligent management of nursing quality, and provides a basis for formulating a unified nursing quality evaluation index system of hepatobiliary surgery. It is of practical significance to improve the nursing quality of ERAS in hepatobiliary surgery.

## 1. Introduction

The ERAS concept first originated in cardiac surgery. ERAS specifically refers to taking evidence-based medicine and effective methods to reduce stress and complications in surgical patients during the perioperative period, reduce the case fatality rate and shorten the hospital stay time, and speed the recovery speed of patients [1]. ERAS not only involves doctors, anesthesiologists, surgical nurses, and other personnel but also includes patients' postoperative nutrition, nursing, rehabilitation, and hospital management and other links. At the same time, it is inseparable from the cooperation of patients and their families. In China, the early application of ERAS is in colon surgery and gastric cancer surgery in Nanjing. The research shows that the treatment of ERAS is effective and safe.

Based on the current clinical medical data, it was found that the incidence of hepatobiliary surgical diseases in China was increasing year by year. Surgery for hepatobiliary surgical diseases was performed through the ERAS concept. It is a relatively effective treatment program for hepatobiliary surgical diseases. Through previous studies, the postoperative body of patients with hepatobiliary surgical diseases is usually in a high score state; patients will experience nausea and vomiting during severe inflammatory reaction. However, ERAS can reduce the emergency body stress response of patients in postoperative care, reduce the occurrence of adverse reactions in patients, and accelerate the patient's condition improvement and recovery. The construction of nursing service evaluation system in hepatobiliary surgery is of great significance for postoperative rehabilitation [2]. Therefore, due to the particularity of hepatobiliary surgical diseases, hepatobiliary surgical care is particularly important.

At present, the quality evaluation of ERAS for hepatobiliary diseases is mainly evaluated through the length of hospitalization and postoperative complications. Some researchers also studied the effect of ERAS implementation in two outcome evaluation indicators in patients and hospitals. However, the lack of research on the index system of ERAS nursing evaluation is conducted. A complete evaluation index system is needed based on the new concept model of ERAS. The development of ERAS requires multidisciplinary team cooperation, and nursing is an important supporting discipline [3]. The perioperative nursing quality evaluation index system based on ERAS theory has high reliability and practicability and can be used as the basis for evaluating the nursing quality of rapid rehabilitation of surgical patients [4]. The established ERAS nursing quality evaluation index system is scientific and reliable and can be used for the quality management of ERAS nursing in general surgery [5]. Therefore, the content of this study is the application value of the new concept of ERAS in the perioperative care of hepatobiliary surgery and the application of ERAS concept in the hepatobiliary surgery care quality evaluation index system construction and empirical research to continue to improve the quality of hepatobiliary surgery care.

## 2. Data and Methods

### 2.1. General Information of Patients

300 cases of hepatobiliary surgical diseases treated in our hospital from January 2019 to December 2020 were randomly selected as the research objects. There were 174 males and 126 females. The average age was 47 ± 6.4 years (25-75 years old). There was no significant difference in general data such as age distribution, educational level, gender, and course of disease (*P* > 0.05). The 300 patients were divided into two groups. The control group was treated with routine perioperative nursing mode, namely, the traditional nursing group. The ERAS nursing group was the observation group, which increased ERAS nursing on the basis of routine nursing. Set up a rapid rehabilitation group with the participation of surgeons, anesthesiologists, nurses, rehabilitation doctors, and patients. There was no significant difference in age, gender, education level, and marital status between the ERAS nursing group and the traditional nursing group. The group was well balanced and comparable. See Table 1 for specific general data of patients.

- Case selection: patients requiring hepatobiliary surgery; conscious, able to fully understand the contents of medical orders, correctly read words, and answer questions; informed consent to this study and voluntary cooperation with this study
- Case exclusion: patients with other serious chronic diseases, other important organ dysfunction, and surgical contraindications before admission; postoperative complications such as bleeding and infection

In order to more intuitively reflect the situation of the patients in the table above, the data in the table were visualized and led to Figures 1 and 2.

In Figure 1, the proportion of patients in the four categories of age, gender, education level, and marital status in the ERAS care group is reflected.

In Figure 2, the proportion of patients in age, gender, education, and marital status in the traditional care group is reflected.

It can be seen from Figures 1 and 2 that there is no significant difference in the general data of the two groups of patients, which can be used in the control test.

### 2.2. Method

#### 2.2.1. Literature Search

Through China HowNet, Baidu Library, VIP, Wanfang medicine, PubMed, MEDLINE, and other well-known databases at home and abroad access to relevant research materials, understand the research status of nursing quality evaluation of hepatobiliary surgery in China, and improve the content of the index system structure of this study. Baidu and other search engines were used to retrieve the national and local standards of nursing quality evaluation and hepatobiliary surgery nursing quality evaluation, as well as the documents related to nursing work, so as to extract important nursing quality indicators.

#### 2.2.2. Questionnaire Survey Method

In this study, the Servqual (quality of service) scale, the pain (VAS) rating scale, and other questionnaires were used to reflect the expected and perceived values of 300 patients on the nursing service quality of hepatobiliary surgery, calculate the nursing service quality score of hepatobiliary surgery in our hospital, clarify the current situation of nursing service quality of hepatobiliary surgery in our hospital, and improve the nursing service quality of hepatobiliary surgery. The grades, scores, and clinical manifestations of the VAS scale are shown in Table 2.

In Table 2, the VAS scale grades the pain levels. The patient evaluated the quality of hepatobiliary surgery in our hospital through the VAS scale.

### 2.3. Statistical Methods

In this study, the statistical data were analyzed by SPSS 20.0 software. Descriptive analysis uses the mean, standard deviation, and coefficient of variation to make descriptive analysis on the indicators. The correlation function formula is as follows:

The “counting (proportion) method” is used to calculate the counting data, and the “mean ± standard deviation method” is used to calculate the measurement data.

The calculation formula of mean and standard deviation is shown as follows:

(1) $$\begin{array}{c} \sigma =\frac{1}{n-1}{\sqrt{\overset{n}{\underset{i=1}{\sum }}\left(x_{i}-\mu \right)}}^{2},\\ \mu =\frac{1}{n}\overset{n}{\underset{i=1}{\sum }}X_{i}, \end{array}$$

where *σ* is the standard deviation, $\bar{x}$ is the arithmetic mean of statistical sequence *x*, *n* is the number of statistical samples, and *x*_*i*_ is the *i*th statistical value in the statistical series *X*.

Bivariate *t*-test was used to compare the data differences, in which the value is *t* value. When *t* < 10.000, it is considered that there is a statistical difference. The smaller the *t* value, the greater the statistical difference. Log value is *P* value. When *P* < 0.05, it is considered to have statistical reliability, and when *P* < 0.01, it is considered to have statistical significance. The calculation formula of *t* value is shown as follows:

(2) $$\begin{array}{c} t_{\text{value}}=\frac{\sum_{i=1}^{n}\left(x_{i}-\tilde{x_{i}}\right)}{\sum_{i=1}^{n}\left(x_{i}-\bar{x}\right)}, \end{array}$$

where ${\bar{x}}_{i}$ is the control value after regression and *t*_value_ outputs results for *t* value. Other mathematical symbols have the same meaning as Equation (1).

## 3. Results

### 3.1. Comparison of Postoperative Nursing Pain (VAS) of Patients

According to the grading, score, and clinical manifestation of the VAS rating scale in Table 2, let the patients score their pain degree according to their own situation. According to the data in Table 3, it can be seen that the score of the ERAS nursing group is significantly lower than that of the traditional nursing group. See Table 3 for details.

In order to more intuitively reflect the postoperative VAS evaluation of the patients in the table above, the data in the table were visualized and obtained in Figure 3.

In Figure 3, it can be seen that the ERAS care group has significantly lower scores than the traditional care group.

### 3.2. Evaluation of the Servqual Scale on Nursing Services in Hepatobiliary Surgery

Servqual scale evaluation is divided into five evaluation dimensions, namely, tangibility, reliability, responsiveness, assurance, and empathy. There are 21 evaluation items. Each item investigates the patient's expectation (*E*) of the nursing service provided and the feeling value (*P*) in the service process. Likert 5-level scoring method is adopted for each item, and the scoring range is 1-5 points. 1 point means very disagree, 2 points means disagree, 3 points means average, 4 points means agree, and 5 points means very agree. Five-dimensional*α*. The expected coefficient is 0.75-0.85, and the perceived coefficient is 0.65-0.78. According to the score difference between the two, the service quality (SQ) is obtained; that is, SQ = *P* (perceived value) − *E* (expected value). There are three cases of total evaluation results: SQ = 0, satisfactory service quality, that is, the actual perception of nursing service is consistent with the expectation of patients; SQ > 0, ideal, that is, the actual perception of nursing service is higher than the expectation of patients; and SQ < 0, dissatisfaction, that is, the actual perception of nursing service does not reach the expected level of patients. Detailed data are shown in Table 4.

In Figure 4, it can be seen from the area chart of Servqual evaluation method for scoring the nursing service quality of hepatobiliary surgery that most of the scoring of nursing service quality of hepatobiliary surgery nursing patients based on ERAS is that the perceived value is greater than the expected value; that is, they are very satisfied with the nursing service quality of ERAS in hepatobiliary surgery, compared with the ERAS nursing group. Although the patients in the traditional nursing group are also satisfied with the quality of nursing service, they are still inferior to the ERAS nursing group. From these two sets of data, we can show that Servqual evaluation method is very valuable for evaluating the quality of nursing service in hepatobiliary surgery, which can be evaluated through different dimensions.

### 3.3. Comparison of Postoperative Adverse Reactions, Satisfaction, and Readmission Rate

There were significant differences in postoperative adverse reactions, satisfaction, and readmission rate between the ERAS nursing group and the traditional nursing group (*P* < 0.05).

In Table 5, the incidence of postoperative complications in hepatobiliary surgical care patients based on ERAS was only 0.64%, the readmission rate was 1.35%, and satisfaction with the overall service of the hospital reached 98.46%. *P* values < 0.05 explain that the services of the ERAS care group are more valuable.

## 4. Discussion

### 4.1. Ethical Argument

The above clinical trial was evaluated and approved by the medical ethics committee. The ethics committee has reviewed the scientificity and ethical rationality of the clinical trial project under the premise of national laws, regulations, and relevant provisions and guaranteed to respect the dignity, safety, and rights of the subjects. Before the start of the trial, fully communicated with the patients participating in the trial, explained the purpose and significance of this study, and signed the informed consent form. Patients have the right to opt out during the study and will deal with the problems of patients in the study in time to ensure the safety of patients. The content of the test shall follow the principle of confidentiality and ensure that the information is not disclosed and not made public.

### 4.2. Significance of Constructing ERAS Nursing Quality Evaluation Index System in Hepatobiliary Surgery

Because of the characteristics of hepatobiliary surgery patients, such as critical condition, complex condition, and many complications, the psychological state and body immunity of patients are relatively poor affected by the disease, and almost all of them have to receive surgical treatment, which increases the workload and difficulty of clinical nursing. Therefore, nursing work should be standardized and scientific. Among them, structural quality is an important part of nursing quality evaluation; that is, structural quality is the basis of quality evaluation. Specifically, it refers to the relatively stable medical support environment in the medical and health service system. Process quality is mainly aimed at the process of nursing service, which refers to a series of standardized behaviors, so it is the focus of nursing quality evaluation. The application of ERAS concept can speed up the postoperative rehabilitation process, save medical resources, and reduce the postoperative pain of patients. Therefore, it is necessary to establish the quality index system of ERAS nursing in hepatobiliary surgery, so as to provide systematic, quantitative, and scientific evaluation standards for the evaluation of ERAS nursing quality in hepatobiliary surgery, which is of great significance to standardize and improve the level of ERAS nursing quality in hepatobiliary surgery.

Establish an ERAS nursing quality evaluation index system for hepatobiliary surgery; we will optimize the nursing quality management mode of hepatobiliary surgery. The scope of the current clinical quality of care standards covers relevant laws and regulations, various nursing technology operations, basic care, and specialty care; however, a set of hepatobiliary surgery evaluation standards with the quality of care as the core is lacking. When the hospital care managers are implementing the quality of care examination, it is often necessary to learn from the comprehensive quality evaluation indicators of hospitals and make your own key content; this makes the evaluation standard of care quality that cannot be unified and increases the difficulty of evaluation. Quality is the first element of hospital management. The quality of care directly affects the quality of medical care. Nursing quality evaluation index system is also an indispensable part of nursing management and remote hospitals to further improve the quality of medical treatment; therefore, the construction of this index provides a more scientific evaluation standard for the evaluation of ERAS care quality in hepatobiliary surgery, it creates conditions for the digital and intelligent management of nursing quality, and it provides a basis for formulating a unified nursing quality evaluation index system of hepatobiliary surgery. It is of practical significance to improve the quality of care of ERAS in hepatobiliary surgery.

## 5. Conclusion

In this study, 300 cases of hepatobiliary surgical diseases treated in our hospital from January 2019 to December 2020 were randomly selected as the current study subjects. Through clinical trials, two groups of study subjects were used: one was the ERAS nursing group and the other was the traditional nursing group. Through the questionnaire survey and access to the relevant research data, statistical data analysis was performed using the SPSS 22.0 software. Metrics were analyzed as descriptive by mean, standard deviation, and coefficient of variation. The Visual Analogue Score (VAS) Hepatobiliary Surgery Nursing Service evaluation form, service evaluation form, postoperative incidence of adverse reactions rate, patient satisfaction, and readmission rate questionnaire were established from the aspects of structural quality and process quality. This study compared the degree of VAS pain through postoperative care. The ERAS care group scored significantly lower than in the traditional care group. The ERAS care group scored significantly lower than in the traditional care group. Nursing patients based on ERAS are very satisfied with the quality of care services. By comparing patient postoperative adverse reactions, satisfaction, and readmission rates, the ERAS care group was significantly better than the traditional care group. By consulting the relevant nursing evaluation system research, supplement and improve the nursing quality evaluation system of this study; moreover, the nursing quality evaluation system is a comprehensive evaluation system of nursing quality from the omni-directional angle of structural quality and process quality. It is also compared with group comparison to highlight the advanced nature and practicability of the nursing quality evaluation system. The later research will further improve and popularize the ERAS nursing quality evaluation index system in hepatobiliary surgery.

## Figures and Tables

**Figure 1:** General data of hepatobiliary patients in the ERAS nursing group.

**Figure 2:** General data of hepatobiliary patients in the traditional nursing group.

**Figure 3:** Postoperative VAS evaluation of patients in the ERAS nursing group and the traditional nursing group.

**Figure 4:** Evaluation of Servqual evaluation method on nursing service of hepatobiliary surgery.

**Table 1:** General information of selected hepatobiliary patients.

General data classification		ERAS nursing group	Traditional nursing group	*t*	*P*
Age	>45	93 (60.0)	90 (62.1)	0.186	0.831
	≤45	62 (40.0)	55 (37.9)	0.204	0.847
Gender	Male	89 (57.4)	85 (58.6)	0.154	0.891
	Female	66 (42.6)	60 (41.4)	0.151	0.846
Degree of education	High school and below	42 (27.1)	39 (26.9)	0.146	0.916
	Junior college and below	78 (50.3)	72 (49.7)	0.102	0.904
	Bachelor degree or above	35 (22.6)	34 (23.4)	0.143	0.881
Marital status	Unmarried	35 (22.6)	30 (20.7)	0.115	0.902
	Married	95 (61.3)	91 (62.7)	0.147	0.824
	Widowed	25 (16.1)	24 (16.6)	0.095	0.964

**Table 2:** Classification, score, and clinical manifestation of the VAS evaluation scale.

Score	Degree of pain
0	No pain
1-3	Slight pain, daily life, and sleep are unaffected and tolerable
4-6	The pain is severe and unbearable, requiring external intervention (oral painkillers and others) and unable to sleep
7-10	Severe pain, passive posture, and obvious autonomic nerve dysfunction

**Table 3:** Postoperative VAS evaluation of patients in the ERAS nursing group and the traditional nursing group ($\bar{x}\pm s$, points).

Item classification	*n*	VAS scores at different time points after operation					
		1 day	2 days	3 days	4 days	5 days	6 days
ERAS nursing group	10	6.3 ± 1.6	3.9 ± 1.3	2.8 ± 0.9	2.4 ± 0.9	1.8 ± 0.9	1.2 ± 0.7
Traditional nursing group	10	3.1 ± 1.3	1.9 ± 1.0	1.3 ± 0.7	1.0 ± 0.8	0.8 ± 1.0	0.7 ± 0.6

**Table 4:** Evaluation of Servqual evaluation method on nursing services of hepatobiliary surgery.

Dimension	Evaluation items	ERAS nursing group			Traditional nursing group		
		Expected value (*E*)	Perceived value (*P*)	Nursing service quality score (SQ)	Expected value (*E*)	Perceived value (*P*)	Nursing service quality score (SQ)
Tangibles	I1	4.89	4.59	-0.30	4.83	4.51	-0.32
	I2	4.78	4.54	-0.24	4.65	4.33	-0.32
	I3	4.86	4.89	0.03	4.83	4.76	-0.07
	I4	4.68	4.55	-0.13	4.75	4.43	-0.32
	I5	4.75	4.80	0.05	4.74	4.85	0.11
Reliability	I6	4.71	4.75	0.04	4.71	4.64	-0.07
	I7	4.64	4.75	0.11	4.76	4.65	-0.11
	I8	4.81	4.85	0.04	4.81	4.82	0.01
	I9	4.72	4.85	0.13	4.75	4.79	0.04
Responsiveness	I10	4.89	4.85	-0.04	4.82	4.81	-0.01
	I11	4.79	4.84	0.05	4.81	4.71	-0.10
	I12	4.74	4.86	0.12	4.64	4.61	-0.03
Guarantee	I13	4.72	4.84	0.12	4.79	4.86	0.07
	I14	4.76	4.92	0.16	4.71	4.82	0.11
	I15	4.78	4.87	0.09	4.73	4.72	-0.01
	I16	4.69	4.84	0.15	4.74	4.72	-0.02
Empathy	I17	4.65	4.75	0.10	4.67	4.71	0.04
	I18	4.79	4.81	0.02	4.81	4.86	0.05
	I19	4.67	4.85	0.18	4.61	4.74	0.13
	I20	4.56	4.76	0.20	4.55	4.57	0.02
	I21	4.64	4.86	0.22	4.62	4.36	-0.26

I1: ward environment, conditions, and other hardware facilities; I2: advanced equipment; I3: the nurse was neatly dressed and dignified; I4: life is convenient during hospitalization; I5: the procedures of admission and inspection are reasonable and convenient for patients; I6: complete all treatment and nursing operations on time; I7: nurses can help patients solve problems in time; I8: nursing records are accurate; I9: timely inform the disease situation, health knowledge, etc.; I10: nurses are on call; I11: the nurse answered the patient's questions enthusiastically; I12: actively patrol the ward and closely observe the changes of the condition; I13: nurses are skilled; I14: nurses are trustworthy; I15: nurses value and respect the rights of patients; I16: in various nursing operations, nurses can ensure the safety of patients; I17: take the patient as the center and arrange the nursing operation time; I18: the nurse was warm and thoughtful; I19: pay attention to the psychological care of patients; I20: to meet the patient needs as much as possible; I21: Be able to handle and improve correctly when receiving complaints from patients.. Dimension: property evaluation of the service scale. Tangibility: evaluate the service facilities, equipment, and instruments of service personnel of the service organization. Reliability: evaluation of service agencies to provide safe and reliable services for patients. Responsiveness: the evaluation service organization is willing to provide timely and effective services for patients. Assurance: evaluate the knowledge and skills of service personnel to make patients have a sense of security and trust. Empathy: evaluate the care and care of service personnel for patients.

**Table 5:** Questionnaire on incidence of postoperative adverse reactions, satisfaction, and readmission rate of patients in two groups.

Item classification	*n*	Incidence of complications (%)	Readmission rate (%)	Satisfaction (%)
ERAS nursing group	155	0.64	1.35	98.46
Traditional nursing group	145	2.07	5.44	83.15
*P* value	—	0.006	0.004	0.003

## Data Availability

The data underlying the results presented in the study are available within the manuscript.
